# NR4A1 retards adipocyte differentiation or maturation via enhancing GATA2 and p53 expression

**DOI:** 10.1111/jcmm.13715

**Published:** 2018-07-25

**Authors:** Dan‐dan Qin, Ying‐feng Yang, Ze‐qing Pu, Dong Liu, Cong Yu, Peng Gao, Ji‐cui Chen, Chen Zong, Yu‐chao Zhang, Xia Li, Xiang‐dong Wang, Yuan‐tao Liu

**Affiliations:** ^1^ Department of Cell Biology Shandong University School of Medicine Jinan China; ^2^ Department of Life Science Qilu Normal University Jinan China; ^3^ Medical Research Center Shandong Provincial Qianfoshan Hospital Shandong University Jinan China; ^4^ Department of Blood Transfusion of Qilu Hospital Shandong University Jinan China; ^5^ Department of Endocrinology Qingdao Municipal Hospital Qingdao China

**Keywords:** adipogenesis, fatty acid synthase, NR4A1, obesity, PPARγ

## Abstract

Nuclear receptor subfamily 4 group A member 1 (NR4A1) is an orphan nuclear receptor with diverse functions. It has been reported that NR4A1, as a transcriptional activator, is implicated in glucose and lipid metabolism. The aim of this study was to investigate the regulatory role of NR4A1 in adipogenesis and explore the underlying mechanisms. Quantitative real‐time PCR and Western blotting were used to analyse the expression of genes involved in synthesis and mobilization of fats in vivo and in vitro. Dual‐luciferase reporter assay was conducted to study the regulatory mechanisms of NR4A1. Our data from in vivo study confirmed that NR4A1 knockout (KO) mice fed with high‐fat diet were more prone to obesity, and gene expression levels of PPARγ and FAS were increased in KO mice compared to controls; our data from in vitro study showed that NR4A1 overexpression in 3T3‐L1 pre‐adipocytes inhibited adipogenesis. Moreover, NR4A1 enhanced GATA binding protein 2 (GATA2) expression, which in turn inhibited peroxisome proliferator‐activated receptor γ (PPARγ); NR4A1 inhibited sterol regulatory element binding transcription factor 1 (SREBP1) and its downstream gene fatty acid synthase (FAS) by up‐regulating p53. NR4A1 inhibits the differentiation and lipid accumulation of adipocytes by enhancing the expression of GATA2 and p53.

**Highlights**

- NR4A1 regulates adipocyte differentiation or maturation.
- NR4A1 inhibits PPARγ expression by enhancing GATA2 transcription.
- NR4A1 partially regulates FAS expression via p53.

## 1 INTRODUCTION

Obesity has drawn more and more attention as it is becoming a severe public health problem. Obesity is a risk factor for many diseases, including type 2 diabetes mellitus, cardiovascular diseases and many others.^1^, ^2^, ^3^ Adipogenesis positively correlates with obesity. So far, the molecular basis and regulatory mechanisms of adipogenesis have not been fully understood.

It is known that obesity is a result of excessive accumulation of body fat,^4^ which is partly due to dysregulated adipogenesis. The differentiation and maturation of pre‐adipocytes are a complex process, in which a series of specific factors are involved. First, CCAAT/enhancer binding protein β (C/EBPβ) begins to express to initiate the differentiation process,^5^ followed by the activation of CCAAT/enhancer binding protein α (C/EBPα) and PPARγ. SREBP1 plays a role in PPARγ activation.^6^, ^7^ At later stage, FAS, fatty acid binding protein (FABP) and other fat synthesis‐related genes are activated,^8^, ^9^ leading to the synthesis of lipids droplets.^10^

On the other hand, lipolysis is the catabolic pathway of fatty acid (FA) cycle. Fatty acids are essential for energy production and the synthesis of most lipids involved in cell structure and cellular signalling. However, an oversupply of FA is highly detrimental.^11^ Factors involved in lipolytic process include adipose triglyceride lipase (ATGL), hormone‐sensitive lipase (HSL), lipoprotein lipase (LPL) and other molecules. To date, some enzymes have been reported to account for complete hydrolysis of triacylglycerol (TAG) molecules in cellular lipid stores: ATGL selectively performs the first and rate‐limiting step hydrolysing TAGs to generate diacylglycerols (DAGs) and non‐esterified fatty acids. HSL is a multifunctional enzyme that is capable of hydrolysing a variety of acylesters including TAG, DAG and monoacylglycerol (MAG). LPL is the rate‐limiting enzyme for the hydrolysis of the triglyceride and very low‐density lipoproteins.^12^, ^13^, ^14^ The fate of obesity formation depends on the balance between the processes of adipogenesis or lipid accumulation and lipolysis.

There are many regulatory factors modulating adipogenesis and lipolysis. GATA2, GATA3, delta like non‐canonical Notch ligand 1 and wingless‐type MMTV integration site family, member 1, are involved in the process of adipogenesis. It was reported that GATA2 bound to PPARγ and inhibits PPARγ expression.^15^ SREBP1 is a transcription factor, which binds to a sequence in the promoter of different genes, called sterol regulatory elements‐1. SREBP1c regulates the expression of genes or enzymes for glucose metabolism and lipid production.^16^ SREBP1c is an upstream molecule of fatty acid synthase.^17^ As reported in other articles, p53 overexpression suppressed the transactivation of SREBP‐1 promoter and the expression of SREBP‐1 downstream genes.^18^, ^19^ In addition, adipokines, including leptin, adiponectin, tumour necrosis factor α, resistin and interleukin‐6, also play a role in regulation of lipolysis.

NR4A1, also known as Nur77, TR3 or NGFI‐B, is a unique transcriptional activator belonging to the orphan nuclear receptor subfamily. NR4A1 expresses in many cell types and mediates diverse biological processes.^20^, ^21^ Recent studies showed that NR4A1 together with two other family members (NR4A2 and NR4A3) played important roles in maintaining cellular energy homeostasis.^22^ It was reported that mice with genetic deletion of Nur77 exhibited increased susceptibility to diet‐induced obesity and insulin resistance.^23^ Some studies showed that NR4A1 had an inhibitory effect on obesity.^23^, ^24^, ^25^ However, the underlying mechanisms remain elusive. In this study, we investigated the role of NR4A1 in adipogenesis and explored the possible mechanisms.

## 2 MATERIALS AND METHODS

### 2.1 Animal study

Both NR4A1 KO mice (generated from C57BL/6J mice) and their comparable wild‐type mice (WT mice) were purchased from the Jackson Laboratory (ME, USA) and were fed ad libitum and maintained in pathogen‐free (SPF) condition. The genotypes of the mice were verified with PCR, in which the primers applied were designed and suggested by the vendor to exhibit the difference between WT and KO (Table 1). Animal experiments were conducted according to the Principles of Laboratory Animal Care established by the National Institutes of Health. All the animal experiment procedures were approved by the Animal Care and Use Committee of Shandong University. The new‐born mice were fed with normal diet for one month and then fed with high‐fat diet for 14 weeks. The high‐fat diet contains 60% fat (6% soybean oil and 54% lard), 20% protein (19.7% casein and 0.3% cysteine), 20% sugar (12.3% maltose dextrin and 6.8% sucrose), provided by Huafukang Bioscience Company (Beijing, China). During this period, the bodyweight of each mouse was measured regularly until the obesity model was successfully generated.

**Table 1:** Primer sequences for PCR or qPCR

For genome identification	
oIMR2060	CACGAGACTAGTGAGACGTG
oIMR6602	CCACGTCTTCTTCCTCATCC
oIMR6603	TGAGCAGGGACTGCCATAGT

Genes	Sequence
For real‐time quantitative PCR	
18S rRNA(+)	CGCGGTTCTATTTTGTTGGT
18S rRNA(−)	AGTCGGCATCGTTTATGGTC
NR4A1(+)	ATGCCTCCCCTACCAATCTTC
NR4A1(−)	CACCAGTTCCTGGAACTTGGA
PPARγ(+)	TGGTGACTTTATGGAGCCTAA
PPARγ(−)	GGCGAACAGCTGAGAGGACTCTG
FAS (+)	GGAGGTGGTGTGATAGCCGGTAT
FAS (−)	TGGGTAATCCATAGAGCCCAG
GATA2(+)	GCCGGGAGTGTGTCAACTG
GATA2(−)	AGGTGGTGGTTGTCGTCTGA
HSL(+)	GATTTACGCACGATGACACAGT
HSL(−)	ACCTGCAAAGACATTAGACAGC
ATGL(+)	ATGTTCCCGAGGGAGACCAA
ATGL(−)	GAGGCTCCGTAGATGTGAGTG
LPL(+)	GGGAGTTTGGCTCCAGAGTTT
LPL(−)	TGTGTCTTCAGGGGTCCTTAG
p53(+)	CCCCTGTCATCTTTTGTCCCT
p53(−)	CCCCTGTCATCTTTTGTCCCT
For DNA molecular cloning	
pGL3‐PPARγ(+)	CCCGGTACCCTCTTCCTCTATCCCGATGGTT
pGL3‐PPARγ(−)	CCCCCTCGAGTCTATGTCTTGCAAAAGATTGGTTG
pGL3‐FAS (+)	CCCGGTACCTGGGAGTGAGAATACACATGGTA
pGL3‐FAS (−)	CCCCTCGAGGATTCCACGCCGCGATCGTA
pGL3‐GATA2(+)	GGGGAGCTCTTCAAACAGGGAGATAATTTTAA
pGL3‐GATA2(−)	CCCCTCGAGACTCCTGCACAGACGTGAAG
For ChIP‐qPCR	
PPARγ(+)	GGAGTCTTTGCATGGTTAGTAACAT
PPARγ(−)	CACCACTGCCCAGCATCCTT
FAS(+)	CGGTTGGGATTCACCAGTCGT
FAS(−)	TACACATACTAGCCAGAGCAGTCC
GATA2‐1(+)	AGAGACATTCACCCAGTGCCAC
GATA2‐1(−)	GTATTCACCATGGGGAGTTCACG
GATA2‐2(+)	CTGGTGCTACAAGGATGTGGTT
GATA2‐2(−)	CATGCTGGCGTGCCCCA

After establishment of obesity model, we carried out different tests or measurements including body fat rate, fat volume, glucose tolerance test (GTT) and insulin tolerance test (ITT) according to the reference.^26^ Epididymal fat was isolated for haematoxylin and eosin staining (H&E staining). We also detected the mRNA and protein levels of NR4A1 in adipose tissues from both WT and KO mice.

### 2.2 Cell culture

The 3T3‐L1 pre‐adipocytes were cultured with high glucose (4.5 g/L glucose) DMEM plus 10% bovine serum (from Gibco), 100 IU/mL penicillin and 100 μg/mL streptomycin at 37°C in a humidified atmosphere with 5% CO_2_. When the pre‐adipocytes reached 100% conference, the medium was replaced with differentiation medium containing 10% foetal bovine serum (from Gibco), 1 μmol/L dexamethasone (from Sigma), 0.5 mmol/L 3‐isobutyl‐1‐methylxanthie (IBMX) (from Sigma) and 10 μg/mL insulin (from Sigma). The day when the inducer was added was considered as day 0 (D0) of differentiation. After two days (D2), the differentiation medium was replaced with fresh medium (high glucose DMEM with serum and antibiotics as described in the beginning of this paragraph) plus 10 μg/mL insulin. After that, the cells were cultured with medium without any inducer and medium was changed every other day (D4, D6, D8). HeLa cells applied to dual‐luciferase reporter gene assay were cultured in high glucose DMEM with 10% foetal bovine serum (from Gibco), 100 IU/mL penicillin and 100 μg/mL streptomycin.

### 2.3 Lentiviral infection and stable cell line selection

Both the Lentivirus encoding full‐length NR4A1 and the control lentivirus were generated by GenePharma as previously described.^27^ 3T3‐L1 pre‐adipocytes were infected with recombinant NR4A1 lentiviral stocks or control lentiviral stocks, and stable cell clones were selected under puromycin drug pressure. NR4A1 overexpression cell lines were designated as OV, and control cell lines were designated as NC.

### 2.4 Antibodies and western blotting

The primary antibodies used to detect mouse proteins were described as follows: rabbit anti‐PPARγ antibody (1:1000), rabbit anti‐FAS antibody (1:1000), rabbit anti‐NR4A1 antibody (1:1000) and rabbit anti‐SREBP1c antibody (1:1000) were purchased from Proteintech Group (Wuhan, China); rabbit anti‐GATA2 antibody (1:1000) was purchased from BioWorld Technology, Inc (St. Louis Park, MN, USA); rabbit anti‐p53 antibody (1:500) was purchased from Santa Cruz Biotechnology, Inc (Dallas, Texas, USA). Mouse monoclonal anti‐β‐actin antibody (1:2000), mouse monoclonal anti‐GAPDH antibody (1:2000) and secondary antibodies (goat anti‐mouse IgG or goat anti‐rabbit IgG) conjugated to horseradish peroxidase (1:5000) were purchased from ZSGB‐BIO (Beijing, China).

Cultured cells or epididymal fat from mice fed with high‐fat diet were washed with ice‐cold PBS and lysed with radio immunoprecipitation assay lysis buffer (RIPA lysis buffer) plus multiple protease inhibitors. The application RIPA lysis buffer contains 50 mmol/L Tris‐HCl (pH 7.4), 150 mmol/L NaCl, 1% Triton X‐100, 1% sodium deoxycholate plus 50 mmol/L NaF, 2 mmol/L EDTA, 1 mM sodium orthovanadate, 10 mmol/L benzamidine, 10 g/mL aprotinin and 1 mmo/L phenylmethanesulfonyl fluoride (PMSF). Vertex and ultrasound were applied for cell lysate. Protein concentration was measured using a BCA Protein Assay Kit (Sangon Biotech). Proteins resolved by SDS‐PAGE under reducing conditions were transferred to PVDF membrane. Then the membranes were blocked and incubated with specific primary antibodies and secondary antibodies. Finally, chemiluminescence signals were detected with a chemiluminescence imaging machine, FluorChem E (ProteinSimple, California, USA).

### 2.5 Quantitative real‐time PCR (qPCR)

Total RNA preparation and quantitative real‐time PCR were conducted as described.^28^ The relative mRNA expression levels were normalized to 18S rRNA. The primer sequences for real‐time PCR are listed in Table 1.

### 2.6 Plasmids construction

Mice genomic DNA was obtained from C57BL/6J liver using an Ezup column genomic DNA extraction kit (Sangon Biotech, Shanghai, China) according to the manufacture's instruction. The promoters of PPARγ (−2000 bp), FAS (−2100 bp) and GATA2 (−2100 bp) were amplified from the genomic DNA with PCR.^27^, ^28^ All the PCR products were sequenced by Sangon Biotech to make sure the promoter sequences obtained were correct by aligning with the sequences from NCBI (GenBank), shown in Table 2. The primers used for amplifying the different promoters are listed in Table 1.

**Table 2:** Promoter sequences

PPARγ GenBank: AH013273.2	AACAAACAGACAAAGGAAGGAAATAATGCCAGCTACAACCCAGGTGGGCTTTGACAACATCATGCTAAGCAAAGGAAACCAATCATACAAGACATTGTATTGTATGAGTCCATTTATAGAAAATATCTAGGGTAGAAAAGTCTATCCAGACAGAAAGTACATGGATGGTGAACCAAGGGCCAATGAGAATGAGGAGGATGAGGAGGAAGTTTCTCTATAGGTTGATAAAAATGTTCTAAAATTAGGTTATGGTGATAATGACACAATTTTGTAAAGAGGCCAAGACTGAATGTGGGGATTTTGAAGATATGGTATTTGAATTTTAGATTATATGAATTATATCTCAATAAAGATGTTAAACTGACACAAGGGATGGGCTGGCCTTAGGAGAATAACAATAAGTTCAAGGCCAGCCAGGACGATATAGCAAGACCTTTTCAAAAAGTTTAATCAAAAGCACAAAACAAAAACCAAACAAAAGTAGATTGAAACTCCTGGGTGAGCAAGAAGTTGGCTACTTACTTACTACATACTTCATACATACATACTTCTCACTGAGTGTGGGATGCTGACCCAAGTCAACATGGCCACTTAATGACAGGCATGGAAATGGAGTCTTTGCATGGTTAGTAACATGGCCTTTAGAGTCCCTATATGAACCTGACCTGTGTCTTATTATTTGAGGACTTAAGAGTGGAAGGATGCTGGGCAGTGGTGGCACATGCCTTTAATCCCAGCCCTTGGGAGGCAGAGGCAGGAGGATTTCTGAGTTTGAGGCCAGCCTGGTCTACAAAGTGAGTTCCAGGACAGCCAGGGCTACACAGAGAAACTGTGTCTCAAAAAACCAAAACCAAAAAAAAAAAAAAAATGTGGAAGGACATGAATCTGTTGATTCAAGCTCTGAACTTTCTTTATAATGTCATACTCACAAATGTCTGGTGAGGATGGTTTGTACCAGAAGAATAAAGAATTCCCTACCTCCCAACAGATAAGGATGCTAAGAGTGGAGAAGCATCTTGAGCAAGAAGCATAATTATAAATTTCCAGAGGCCAGTGCCTCCTAAAGGAGAGCAAAACATAGAGCAAGGTCTTCATCATTACGATTGGAAAAGGATAAAAGAACGGCCTTTGGTGTCCTGGACACTGCAAGCTTTCTGAATGTGAATCTTTAGGACAGATCATGACTGTGAGAGCTGAAAGAGTGCAAGAAAAGGAACTGTCTATCATGTGGGCTTCAGGCTCCCGAGGCAAGAAGCTCCAATAGTCTAACTTAAAAACAAGAGATTCTCAGGCCCTCTCCACCCTATGTGTAAGGTCTCCTATGTAAGAAATGGTGCTAAAGAATTTTAAAAAGCCAGTGAACAAGGTTAACAAATAGTTTGAAGGCAGGAGAGATTGCTCAGCGGTTAGGAACACTTTGTGTTCTTCCAGAGGACCCTTGTTCGGTTCCCAGCACCAACCACCTGTAACTCCAGCTCCAGGGGAGCCCACACCTCTCCCTCCGTTCACGTGCATACACACACAATTGTTTTTTAAAAGGAAATTAAATGATTAGCACTAAAGTCTGTTGATTAAGGCATTCGCCTTCATAACATTCTGAGATTAAAAATAAAAATAAAACTGAGATTAAAAATAAAAAGAAAAAAAGAAAAAAGGGAGATCCTAAATTCACTTAATTCATATAAATATATATATGGGTGTGTATCTATTATATATCATATATCATATATATGATATATAAATATATGTTATGTATGATATATAAATATATATGGTATATATATAGAGAGAGAGATGAAAAGCACATCTAGGAAAAAAACAAACTTCTCCATGACAGACATGGACATGGACATCGGTCTGAGGGACACGGGACCTTCCTGGGTCGCCTCCCAGCGGCTGTGAGGAGCAAGGCGGCCAGGTAACCAGCGCACGGCGCCGGGCGCGGGAGGGCCACGCGGGCCTCGTGGGCGCCGGCCTCCGGGTGCGGGCGCGGGGCCTCC
FAS GenBank : AL663090.15	CATCTGTTTGGCCTGTGAAGTTGTCTGTCTTGTCCTACTTGGGGAATGCAGGCTGGATCCTGGGCTGGCCTCTGCCCCCTGCCTGTCACCACCCACAGCCACTGTGCACTCGCCCTGTCGGTGACACTGTCCTCCAGAGCCTGGTGGGCAGAATAGAGTGGCCACCTGCAAAGTATGTCCCCAAGGAACACTGTATGAGAGGTCCTCCCGGGAGCATGGGCCTGGCCACCCAGAGGCCCAGTCTCGGAACCAGACCCATCTGCCTACTGAAAACCTCATGAGACCTGCCTGACCACTTCCTGTCCATAGCATGACTTAAAGAGGCCCATGGCCTTAGCCTTGCTGGGTATCAGACACACAGGGCTGCAGGGTCCAGGCAGCTCCCAGGTCCAGGTTGTTGTGTGTCCTTGACTAATCATGTGACTCTTGCAGCTTCATTTTTGCATCTCTGTGTGTAAAATCCTGACAGTGATTCCAGGCTGGCTGGCTCACATGGTGGGCCATCACAACATTACAGGGAAGCCCACACTCAGTAATGTGGTCTTGGATGCCAGTTGAATAACTCAGGCCTAGGTAGCAGACATCTGCAGATCACTCCTGCTGTGGGTCTGTAGTAGGTAGCTCTCAAGGTGCATATGCAAAGAGAGAGCCATAGGATGCTTTTACAAGAGCCCACCTAGGTACACTGTGCTGTTTTCACGACTGGCAGGGGCCATGGCAGGCCATCCTGACGTGGCTCTCTCATATCCACATCTGGCAATCCACTTTGTTTGTCACGTGTTTCTGAGATGTAGCCATGCAACTTCCTTTGGTGAAAAGATGATCAGAGAAGTTTGCTCTGCCCTCAGCATCCTGCTCTGTGCACGGCCCAGACTCTGCATCCCTGGGTTACATCTCCTCCAGCTGAGACCCTGACAGCTGCAGAGGGCAGAGCTCTGCTGACCACTTAGGGTTGGCCAGCAGCCTGGCCAGTGAGAAGGCAAACATGACCTATCTCAAGGCACCAGGAGCTGGGGTGGGACTGCTCTGGCTAGTATGTGTACAGGCCTTTTGTAAAACTTTCCTAGGCTGGCCCTGAAACCCAAAGACACCCACAAAGGCATAGGGGCAAAATGGGAGAGCTTGGGGGCAAGCCAGCTTATGGGCAGAATACACCTGCCAGTCCTATAGGCTGCCCTTCAGGGTCCCTGCTTAGCCTCCTTCCACAGAAAGCCTGGGTGGATAGCCAAGTTGGAGAAGCTAGAAGCCAGGGTTGACAAGCAAGGCTCTGAGGCTCTGGCTTTTGCTATAGACTTGCAGTCAAGGACCACTGACACTAGCCCCCTTCCCCCTCCCCCCCACTCCCGGGCCATTACCCCATAAGGAGGTCAGTCTTAGTGGCCTGGGCCTGTAGTGGAAGGACAGGAGGGAAGGGAACAACCTCTCTAGGCACTCAAGGGACCCAACCCTGAGAAGTCTGTGTCTTTTTGGACGGTGAGTTTTGTCATCCCCCGCCCCCAAATTCGATAACCCTTTGAAAAGAGGAATTTAAAGGGAGGGAGGGAGAGGGTCCCGGAAACTCAGGGAGGCGCGCAGCAGCTCCTTTGTTCCCACCAGGCGGGGGAGGGGTGGTATCCCGCTCGCCAGATGGCCGCGCCTGGACACTGAGCGGACTCCGGAGGCCGCCACACGCGCCCGTCAGTGTTCCCTATCCTGCCTACTGCTCCCGTCCCTGCCCGCATCCTGGTCTCCAAGGTGGCCACAGAGGGTGGGAGTCCGAGAAAGCTGGGCCACGATGACCGGTAGTAACCCCGCCTGAGGCGCCCTCCGCCAGGGTCAACGACCGCGCTTGCGCGGGGGCCCGCGAAGTGCTTTGCCGCTGTTGCCGGCCCATCACCCTATTGCCTAGCAACGCCCACCCGCGCGCCGCCATTGGGCCACCGAGAACGGCCTCGGTGTCCAATTGGTTTCGATGTGGAGCAGGCCACGCCCCTCGGTTCCGCGCGCGCTACGATCGCGGC
GATA2 GenBank: AB007371.2	TCCCCCTCCCACAGACATACAGAAAGTGCCAGAGTAAATGGCACCCCGGGGCTCCCCTGGCTGCCTGCCCTGATGGTTAGGGAAGGTGCGGCTGGCTAGGGAGCCTGCAGGGTACACATACTGTCTCCACACCCCTCCCCTTCCAGACATAGAGTAACCCTGGCTACAGAAACACAGATCCAGGATGGAAGGATGGTCAGAGGTGCCCACCCCTCAAGCATGGCCACAACCATCAAGCTCCCCCCCAAAAAAAACCATCAGTGTCAACCAAAGCAATAGCTCCGCAGACATATGTTTGCCCCCATCTACCTTCAGCTCCAAGTTAGACATCAACACCTGCCATTAAGACAAGCTAGCCCCGAGTGGCAGGACATGCCTTTAATCCCAGCACTTAGGAGGCAGAGGCAGGCATATCATTATGAGTTCCAGGCCAGCCATGGTGACATAATAAGACCTTGCTTTAAAATAACTGTATGGCCACACAACTGTATGGCCTCAGATACACAGACCCCCCCCCCACTGCCCCAATGAATTAATACAATTGTCAGTAAGTATCCAGACACATTGCAAACATCTCACTTGTGTACACACACACACACACACACAGAGAGAGAGAGAGAGAGAGAGAGAGAGAGAGAGAGAGAGAGAGAGACTATTAAAGATGGAAACAAATGCATGCCTAGATATATACACAAATGTACAAAGGTATTACACTGATTAAGACATACTTATAGATACCGACTGCCTATCACATGATTCCTGAAGCTGATGGTCTATCTCAGAGAGATAGGTGCAGATGCAGAGACATTCACCCAGTGCCACAGATACTCTCTTGTGTGCATTTGTGGGGCCACACACTGGTAGCAGTCGTGCTGTGACCTTCAACCCAATACAAATGCTTAGGGACACCCTTAAGTTTTGCAAACACTCCCGTGAACTCCCCATGGTGAATACATAGGCCACTGGGCACATAAACTGAGCTGCGTGTAGACGGTACATACACAAAGCAAAAGATTCAGAAAGATCCAAAACATCTGGTGCTACAAGGATGTGGTTGCAGGGACTGACCTACTCCCTGGATGGGGCACGCCAGCATGCAAGGTCTTTCCGAGAAGAGAGAGTCTGTAGAGTTCTTTGAATTTCTCAGAGGGGTTTAGGATAATATAAGGAATGAATTCTCATTGCTATCTAGCTCAGGTGCCTCCTTAAGTTGTAGACTGCCACGAGGCTTCCTCCCTTCTAAGGACAAACGTTTTGCTCTTCTTGTGGCTCTCTCTGATGCAAAAGGTTCACCAAGAATGGGCCAGAAACTCCATTCCTAAAATGCTTCTGAGTTGGGAACTGGCATCTGTGGGGAAGAATGTGGGAAAGCATCTACACATAGCCAAATGTGCAGGAAGGATGGGAGGTGTGTGTGTGTGTGTGTGTGTGTGTGTGTGTGTGTGTACATTATATCTATATGTGCACCGGTGTTTGTGTGCCAGAAAGCCCCTGTCTGGGGACATCTACACAGTGCATAACGGTGTGTCTGAAAGGAGGGGCAGGTGTCTGTGTACTTGCTTGTGAGGGAGAGTCTCAAAAGAGAGACATCGCAGGCTTTCAGAGATTACATCCCTGAGAGCAGAAGTGCTTGCGTGGCCCTGAGAAGGCGGGAGTGGCCTGCAGGGTGTGCGCGCCTCGACTGACTAGTGGCCCAAGCCTGGCCAGCCCGGCGGCTGGACCAGGCAGACAGGGCGCAGAGCCCGGGCACCCTCCTGCCCCCCTGCGGCGTTCCCTCCCCCCCTCGAAGTGATGTCGAAATAAAAAGCTGCCGCTCTGCGGCCGGGAACCGAGAGACAGCCAGAACCAAGAGAGGTGGCCAGGCCAGCGGGGCGGTAGCTCACTGCTCAGGTCTCCCTGGCCTAAGATCACCTCAACCATAGCCGGTCTCGGGGGACAAAAGCGGCTGCCTGCGCGACGAGCTTGCGTTCCGCGCCGCGGGGGCCCCACTGGTGACCGCC

### 2.7 Dual‐luciferase reporter gene assay

HeLa cells were seeded into 24‐well plates for 24 hours, thereafter, they were transiently transfected with a luciferase reporter plasmid (pGL3‐PPARγ, pGL3‐FAS, pGL3‐GATA2 or pGL3‐basic) plus the thymidine kinase promoter‐Renilla luciferase reporter plasmid (pRL‐TK) using TurboFect Transfection Reagent (Thermo Scientific). At 24 hours post‐transfection, the luciferase activity in each well was measured with a dual‐luciferase reporter assay kit (Beyotime Institute of Biotechnology, Shanghai, China) according to the manufacturer's instructions.

### 2.8 Chromatin immunoprecipitation assay

Adenovirus encoding NR4A1‐haemagglutinin (HA) (Ad‐NR4A1‐HA) or Control adenovirus (Ad‐GFP) were amplified, purified and enriched according to standard technology.^29^ 3T3‐L1 cell was infected with NR4A1‐HA adenovirus (AD‐NR4A1) or control adenovirus (AD‐GFP) for 48 hours. Then cell samples were applied for Chromatin immunoprecipitation assay (ChIP) assay with a commercial available kit (Beyotime Institute of Biotechnology, Shanghai, China) according to manufacturer's instructions. The anti‐HA tag monoclonal antibody (Santa Cruz Biotechnology, Inc, Dallas, Texas, USA) was applied for immunoprecipitation. The precipitated DNA fragments were purified with a universal DNA purification kit (Tiangen Biotech, Beijing, China). Finally, qPCR was employed to check the specific DNA sequence from the purified DNA fragments. Sequences of all primer pairs used in this study are listed in Table 1.

### 2.9 Statistical analysis

Statistical data were expressed as mean ± SE. Comparisons were performed by one‐way analysis of variance (ANOVA), followed by the Newman‐Keuls test using SPSS 17.0 software package. A value of *P *< .05 was considered statistically significant.

## 3 RESULTS

### 3.1 NR4A1 knockout mice are confirmed with PCR and Western blotting

The genotypes of mice were confirmed by ordinary PCR, qPCR and Western blotting. The mouse tail was used for DNA extraction and PCR amplified by three primers as suggested by the Jackson Laboratory (oIMR2060: 5′‐CACGAGACTAGTGAGACGTG‐3′; oIMR6602: 5′‐CCACGTCTTCTTCCTCATCC ‐3′; oIMR6603: 5′‐TGAGCAGGGACTGCCATAGT‐3′.). After the PCR cycles were completed, the DNA products from the PCR were separated by agarose gel electrophoresis. KO mice exhibited a target band about 350 bp that was amplified from a pair of primers named as oIMR2060 and oIMR6602, while WT mice exhibited a target band about 180 bp that was amplified from a pair of primers named as oIMR2060 and oIMR6603 (Figure 1A). qPCR results showed that WT mice had higher mRNA level of NR4A1 (Figure 1B), Western blotting results showed that KO mice had less NR4A1 protein signal compared to WT mice (Figure 1C).

**Figure 1:** Analyses of NR4A1 knockout mice. A, Confirming the genotype of KO mice. The DNA from the mouse tail was extracted and subjected to PCR and electrophoresis according to the method provided by Jackson Laboratory. KO mice exhibited a target band about 350 bp that was amplified from a pair of primers named as oIMR2060 and oIMR6602, while WT mice exhibited a target band about 180 bp that was amplified from a pair of primers named as oIMR2060 and oIMR6603. B, The relative NR4A1 mRNA levels in mouse epididymal fat both from WT and KO mice. C, The relative protein levels of NR4A1 in mouse epididymal fat both from WT and KO mice. The data show the means of three independent experiments. **P < .01, ***P < .001

### 3.2 NR4A1 knockout mice (KO) are more inclined to develop obesity under high‐fat diet

KO and WT mice of similar age (within 1 week's difference) were used for experiments. These mice were fed with normal diet for a month. Afterwards, the mice were fed with high‐fat diet for 14 weeks, and the mice bodyweights were measured regularly (Figure 2A). Results from H&E staining showed that the size of cell surface area from KO mice was much larger compared to that of WT mice (Figure 2B). By comparison of the percentage of their body fat and fat volume, we confirmed that KO mice fed with high‐fat diet were more likely to gain weight (Figure 2C and D). GTT and ITT were conducted to detect the insulin sensitivity in different mice. GTT results showed that KO mice had prolonged and higher blood glucose levels after glucose injection when compared with WT mice (Figure 2E). ITT results showed that blood glucose levels of WT and KO mice were both reduced after insulin injection, but there was no significant difference in blood glucose levels between KO and WT (Figure 2F).

**Figure 2:** High‐fat diet inducing obesity in mice. (A) Bodyweight changes in WT mice and KO mice during 14‐wk high‐fat diet feeding. (B) Analysis of fat cells size in white fat with H&E staining. (C) Measurement of the size of mouse epididymal fat. (D) Detection of body fat rate in WT and KO mice. After 14 wk of high‐fat diet feeding, WT and KO mice were tested for GTT (E) and ITT (F). The data show the means of three independent experiments, *P < .05, **P < .01, ***P < .001

### 3.3 PPARγ and FAS expression is increased in adipose tissues from KO mice

We collected epididymal fat tissues to analyse the expression of obesity‐related genes implicated in fat synthesis and degradation. The mRNA levels of lipolytic genes, including HSL, ATGL and LPL in the fat tissues from KO mice showed no significant differences compared to those of control (WT) mice (Figure 3A). In KO mice, the expression levels of C/EBPβ, adiponectin, FABP4 in adipose tissues were similar to those in WT mice (Figure 3B and C). We also detected the expression of C/EBPα, another marker of adipogenesis, in adipose tissues of WT and KO mice, and found no significant difference (data not shown). However, the protein and mRNA expression of lipid synthesis‐related genes, PPARγ and FAS, were increased in adipose tissues of KO mice (Figure 3D, E and F).

**Figure 3:** NR4A1 impacting the expression of PPARγ and FAS in KO mice. Mice were fed with normal diet for one month after birth and then fed with high‐fat diet containing 60% fat for 14 weeks. And their foetal epididymal fat was harvested after 14 wk of high‐fat diet. A, qPCR analysis of HSL, ATGL and LPL in mouse epididymal fat both from WT and KO mice. B, Relative mRNA levels of C/EBPβ and adiponectin in mouse epididymal fat. C, Relative protein levels of FABP4 in mouse epididymal fat. D, Relative protein levels of PPARγ in mouse epididymal fat. E, Relative protein levels of FAS in mouse epididymal fat. F, Relative mRNA levels of PPARγ and FAS in mouse epididymal fat. The data show the means of three independent experiments, *P < .05, **P < .01, ns, no significance

### 3.4 NR4A1 inhibits the adipogenesis of 3T3‐L1 pre‐adipoctes

During adipogenesis, NR4A1 expression profile showed a similar trend with PPARγ and FAS (Figure 4A). To clarify the role of NR4A1 in adipogenesis, 3T3‐L1 cell lines overexpressing NR4A1 (OV) and control cells (NC) were used. After the cells were induced to differentiate, Oil Red O staining was used to examine the level of adipogenesis. We found that NR4A1 overexspression reduced the differentiation rate of 3T3‐L1 pre‐adipocytes (Figure 4B). During the period of induced adipogenesis, cells were harvested and protein samples were collected at different time‐points, and Western blotting was conducted to detect protein expression levels. Results showed that NR4A1 inhibited the protein expression of PPARγ and FAS during adipogenesis (Figure 4C).

**Figure 4:** The possible role of NR4A1 in adipogenesis. The initial day to add the inducer was regarded as D0. 3T3‐L1 Cells were cultured continuously for 8 days and harvested every other day. (A) Western blotting analyses of NR4A1, PPARγ and FAS during 3T3‐L1 differentiation. The overexpression cell lines of NR4A1 (OV) and its control (NC) were obtained by lentivirus infection and selection under puromycin drug pressure. They were induced for adipogenesis and stained with Oil Red O to monitor the degree of differentiation (B). (C) The relative protein levels of PPARγ and FAS during differentiation period between NC and OV cells. The data show the means of three independent experiments, *P < .05, **P < .01, ***P < .001

### 3.5 The possible mechanisms of effects of NR4A1 on adipogenesis

Overexpression of NR4A1 reduced the expression of PPARγ and FAS, and both PPARγ and FAS have putative NR4A1 binding sites on their promoters (Figure 5A). We constructed the luciferase reporter plasmids containing 2000 bp promoter of PPARγ or 2100 bp promoter of FAS to explore whether NR4A1 had effects on the transactivation of these two promoters. The luciferase assay results showed that NR4A1 had an inhibitory effect on PPARγ transcription, but had no effect on FAS (Figure 5B). ChIP‐qPCR results showed that NR4A1 had no direct physical association with PPARγ or FAS (Figure 5C).

**Figure 5:** NR4A1 regulating the transcription of adipogenesis‐related genes. A, Putative NR4A1 binding sites (a putative NBRE) in promoters of PPARγ, FAS and GATA2. B, Dual‐luciferase reporter gene assay for PPARγ, FAS and GATA2 promoters. C, ChIP‐qPCR was exploited to analyse the physical association between NR4A1 and the promoter region of PPARγ, FAS or GATA2. The data show the means of three independent experiments, *P < .05, **P < .01, ***P < .001

However, NR4A1 as a transcriptional activator inhibited the adipogenesis of pre‐adipocytes, we speculated that NR4A1 might activate the expression of some specific inhibitory factors, which in turn inhibited the expression of essential factors for adipogenesis. In some previous studies,^29^ GATA2 was reported as a transcription factor that inhibited PPARγ transcription by binding to its promoter. We found that NR4A1 was able to enhance the transactivation of GATA2 promoter (Figure 5B). Furthermore, we found that NR4A1 was able to bind to the promoter of GATA2 by means of ChIP‐qPCR test. Then we studied the NR4A1 binding site on GATA2 promoter and figured out that NR4A1 bound to one putative binding sequence between −1125 bp to −1120 bp (GATA2‐1) on the GATA2 promoter but did not bind to another putative binding sequence between −936 bp to −931 bp (GATA2‐2) (Figure 5C). GATA2 expression was decreased in adipose tissues from NR4A1 KO mice (Figure 6A and B) and increased in OV cells during adipogenesis in vitro (Figure 6C).

**Figure 6:** NR4A1 modulating GATA2 expression. A, Relative protein levels of GATA2 in mouse epididymal fat. B, Relative mRNA levels of GATA2 in mouse epididymal fat. C, Relative mRNA levels of GATA2 in the process of adipogenesis differentiation in both NC and OV cells. The data show the means of three independent experiments, *P < .05, **P < .01, ***P < .001

As NR4A1 showed no direct effect on FAS, so we explored the upstream genes of FAS, especially, SREBP1c. Our data demonstrated that the expression of SREBP1c was also reduced in OV cells (Figure 7A). Then we examined the expression of some inhibitory proteins for SREBP1, including AMRK and ATF6, but none of them was positively correlated with NR4A1 expression (data not shown). As p53 was also reported as an inhibitory protein for SREBP1c expression,^30^ we therefore checked the expression of p53. Our data showed that the expression of p53 at both protein (Figure 7B) and mRNA levels (Figure 7C) in adipose tissues of KO mice was reduced.

**Figure 7:** NR4A1 modulating FAS pathway. A, Relative protein levels of SREBP1c during adipocyte differentiation. B, Protein expression of p53 in mouse epididymal fat. C, Relative mRNA levels of p53 in mouse epididymal fat. D, A model for possible roles of NR4A1 in inhibiting adipogenesis and controlling bodyweight. The data show the means of three independent experiments, *P < .05, **P < .01, ***P < .001

## 4 DISCUSSION

In this study, we further confirmed that NR4A1 knockout mice were more likely to gain weight.^18^ Moreover, we found that NR4A1 overexpression inhibited adipogenesis in 3T3‐L1 pre‐adipocytes. In vivo, it has been reported that NR4A1 had the effects on glucose and lipid metabolism in liver 31, 32 and muscles.^30^, ^33^ Studies have shown that NR4A1 knockout mice fed with high‐fat diet were more likely to develop obesity compared to WT mice.^23^ In consistency with previous study, our results also showed that NR4A1 KO mice fed with high‐fat diet were inclined to develop obesity compared to WT mice. We examined the morphological changes of adipocytes and the expression profiles of genes associated with adipogenesis or lipid accumulation in KO mice. We found that KO mice fed with high‐fat diet resulted in increased size of adipocytes or increased fat volume in comparison with WT mice, while the expression of PPARγ and FAS in the adipose tissues from KO mice was increased compared to that from WT mice. PPARγ and FAS are important factors for adipogenesis, in particular FAS is an essential enzyme for lipid synthesis or lipid accumulation. The above data indicated that NR4A1 might have inhibitory effects on adipogenesis and lipid accumulation.

In vitro, it was reported that NR4A1 would inhibit adipogenesis of 3T3‐L1 adipocytes.^24^, ^34^ We found that overexpression of NR4A1 in 3T3‐L1 pre‐adipocytes reduced adipogenesis. Pols et al^32^ found that NR4A1 down‐regulated SREBP1 and its downstream genes including mitochondrial glycerol‐3‐phosphate acyltransferase, acetyl‐CoA carboxylase‐α in hepatic lipid metabolism. Maxwell et al suggested that NR4A1 would modulate the expression of adiponectin receptor 2, uncoupling protein 3 and protein kinase, AMP‐activated gamma 3, to enhance lipolysis; therefore, NR4A1 could negatively regulate adipogenesis,^24^ but the mechanism remains elusive.

Our data showed that the expression of PPARγ and FAS was significantly increased in NR4A1 KO mice. Consistently, overexpression of NR4A1 in 3T3‐L1 cell line reduced the expression of PPARγ and FAS, suggesting that NR4A1 possibly impacts both adipogenesis and lipid accumulation. Furthermore, our data showed that NR4A1 seemed to have no apparent effect on lipolysis as NR4A1 did not change the expression of lipolysis‐related genes. We searched the promoter sequences of PPARγ and FAS and found that both PPARγ (from −1339 bp to −1334 bp) and FAS (from −1014 bp to −1009 bp) had NR4A1 putative binding sites (5′‐TGACCT‐3′) (Figure 5A). Results of luciferase assay showed that NR4A1 inhibited the transcription of PPARγ, but had no effect on FAS. As a transcriptional activator, NR4A1 usually binds to a promoter and enhances its transactivation. Our data showed that overexpression of NR4A1 reduced the transactivation of PPARγ, indicating that NR4A1 might down‐regulate PPARγ expression indirectly. We thus looked into the negative regulators of PPARγ. It was reported that GATA2 bound to the promoter of PPARγ and inhibited PPARγ expression.^15^ Then we searched the promoter sequence of GATA2 and found that there are two NR4A1 putative binding sites in this sequence. The luciferase assay data showed that overexpression of NR4A1 in 3T3‐L1 pre‐adipocytes enhanced the transactivation of GATA2 promoter. Furthermore, we confirmed that NR4A1 had physical association with GATA2 promoter by exploiting the ChIP‐qPCR techniques, but no physical association with PPARγ promoter. There are two putative NR4A1 binding sites in GATA2 promoter (from −2100 bp to 0 bp). We further narrowed down the effective binding site (from −1125 bp to −1120 bp) rather than another one (from −936 bp to −931 bp). We proposed that NR4A1 might inhibit adipogenesis through up‐regulation of GATA2, which in turn could inhibit PPARγ expression.

It was also reported that SREBP1c positively regulated the transcription and expression of lipogenic enzymes such as fatty acid synthase. It was a key transcriptional regulator of triglyceride synthesis.^35^ In this study, overexpression of NR4A1 in 3T3‐L1 cells resulted in reduced expression of SREBP1c. We searched some related research articles and found that p53 was reported to have an inhibitory effect on SREBP1c expression.^18^, ^19^ Our data exhibited that NR4A1 overexpression suppressed the expression of the SREBP‐1c and its downstream FAS. While knockout NR4A1 resulted in reduced p53 expression, therefore, NR4A1 might indirectly modulate the expression of SREBP‐1c via p53, then hinder excess fat accumulation in adipocytes.^18^, ^19^ It has been reported that NR4A1 could either enhance DNA‐dependent protein kinase to increase p53 transcription activity 36 or to cause mouse 3T3 cell double minute 2 (MDM2) to separation from p53, thus to protect p53 from MDM2‐mediated ubiquitination and degradation.^37^ Herein we confirmed the presence of p53 in adipose tissue and found that p53 expression was reduced in adipose tissues of KO mice compared to WT. Based on these findings, we proposed that NR4A1 might indirectly reduce the expression of FAS by up‐regulating p53 expression and subsequently down‐regulating SREBP1c expression. Therefore, we proposed that NR4A1 might regulate adipogenesis and bodyweight via two possible pathways as shown in Figure 7D.

In summary, this study demonstrated that NR4A1 inhibits adipogenesis or adipocyte maturation. NR4A1 directly up‐regulates GATA2 expression, which reduces the transcriptional expression of PPARγ; and NR4A1 indirectly down‐regulates SREBP1c and subsequently down‐regulates FAS through p53.

## CONFLICT OF INTEREST

The authors confirm that there is no conflict of interests.
